The article "From Twitter to Aso-Rock: A sentiment analysis framework for understanding Nigeria 2023 presidential election" was published in 2023. Journal: Heliyon.

# From Twitter to Aso-Rock: A sentiment analysis framework for understanding Nigeria 2023 presidential election

**DOI:** 10.1016/j.heliyon.2023.e16085

**Published:** 2023-05-12

**Authors:** Olusola Olabanjo, Ashiribo Wusu, Oseni Afisi, Mauton Asokere, Rebecca Padonu, Olufemi Olabanjo, Oluwafolake Ojo, Olusegun Folorunso, Benjamin Aribisala, Manuel Mazzara

**Affiliations:** a Department of Mathematics, Morgan State University, USA; b Department of Computer Science, Lagos State University, Ojo, Lagos Nigeria; c Department of Mathematics, Lagos State University, Ojo, Lagos Nigeria; d Department of Philosophy, Lagos State University, Ojo, Lagos Nigeria; e Department of Theatre Arts, Ahmadu Bello University, Zaria, Nigeria; f Department of Computer Science, Oduduwa University, Ile-Ife, Nigeria; g Department of Computer Science, Federal University of Agriculture, Abeokuta, Nigeria; h Institute of Software Development and Engineering, Innopolis University, Innopolis, Russia

**Keywords:** NLP, NLU, Twitter, Sentiment analysis, Opinion mining, Nigeria, Election, Machine learning, BERT, LSTM, SVM

## Abstract

**Introduction:**

Social media platforms such as Facebook, LinkedIn, Twitter, among others have been used as tools for staging protests, opinion polls, campaign strategy, medium of agitation and a place of interest expression especially during elections.

**Aim:**

In this work, a Natural Language Processing framework is designed to understand Nigeria 2023 presidential election based on public opinion using Twitter dataset.

**Methods:**

Two million tweets with 18 features were collected from Twitter containing public and personal tweets of the three top contestants – Atiku Abubakar, Peter Obi and Bola Tinubu – in the forthcoming 2023 Presidential election. Sentiment analysis was performed on the preprocessed dataset using three machine learning models namely: Long Short-Term Memory (LSTM) Recurrent Neural Network, Bidirectional Encoder Representations from Transformers (BERT) and Linear Support Vector Classifier (LSVC) models. This study spanned ten weeks starting from the candidates’ declaration of intent to run for Presidency.

**Results:**

The sentiment models gave an accuracy, precision, recall, AUC and f-measure of 88%, 82.7%, 87.2%, 87.6% and 82.9% respectively for LSTM; 94%, 88.5%, 92.5%, 94.7% and 91.7% respectively for BERT and 73%, 81.4%, 76.4%, 81.2% and 79.2% respectively for LSVC. Result also showed that Peter Obi has the highest total impressions the highest positive sentiments, Tinubu has the highest network of active friends while Atiku has the highest number of followers.

**Conclusion:**

Sentiment analysis and other Natural Language Understanding tasks can aid in the understanding of the social media space in terms of public opinion mining. We conclude that opinion mining from Twitter can form a general basis for generating insights for election as well as modeling election outcomes.

## 1 Introduction

Forecasting and analysis of election results have gained a wide popularity in the field of political methodology [1], a subfield of political science and political analysis concerned with the study of quantitative and qualitative approaches used to understand politics and political systems [2]. These methods often combine statistics, mathematics and formal theory for the understanding of politics. Election results have usually been predicted in the past using analytical and statistical techniques where the methodology relies on surveys and qualitative methods, and analyzing political party manifestos while observing the trends in the mainstream media [3,4]. With an increased contest and opposition in the government, particularly in nations with multi-party system like Nigeria [5,6], it has become more difficult but interesting to predict elections.

The power of social media and how greatly it has been established to affect elections and electoral systems motivated this study. The influence of social media on elections became noticeable first in the early year 2000 [6]. In his first presidential campaign, Barack Obama made use of social media to mobilize the public and win the 2008 election. Statistics revealed that 74% of internet users—or 55% of the adult population—looked for election news online during Obama's first campaign. Another famous example is when Beto O'Rourke came dangerously close to unseating Senator Ted Cruz in 2018. The 2018 Texas Senate race broke the record for the most money spent in a U.S. Senate election, according to the Center for Responsive Politics, spending $93 million, a large portion of which was raised from and used for social media events and advertisements. The social media is, no doubt, a key tool to understanding and analyzing public political opinion and predicting election outcomes.

Before and after the social media revolution, surveys have been used frequently to identify opinions prior to elections; however, this approach has been limited by the difficulty in constructing an appropriate sampling procedure, hence making it difficult to obtain a representative sample of political viewpoints. Social media platforms such as Twitter, Facebook, Reddit and Instagram have helped in some way to overcome the “systematically inappropriate” sampling procedure in survey studies and have been the prominent tools of political campaigns and activisms during elections. The recent advancements in the fields of Natural Language Understanding (NLU) and Natural Language Processing (NLP) have improved the reliability of prediction models built for unstructured and unsupervised dataset [7]. The social media has radically upended the traditional campaign norms and tactics in national elections vis-à-vis its volume, velocity, scope and tactics of use [8,9]. Studies also showed that even if it cannot be categorically said that social media singlehandedly elected Donald Trump, his social media campaign strategies changed the way social media will be used in elections in the future [9,10].

There has been a growing interest in the use of NLP and other artificial intelligence techniques to predict election results in recent years with social media datasets. These techniques include sentiment analysis and topic modeling in addition to more advanced models that incorporate deep learning and fundamental statistical techniques. Two important aspects of NLP are sentiment analysis and opinion mining, which aid in classifying and investigating the behavior and approach of social media users with regards to brands, events, companies, customer services as well as elections. There are algorithms for automating the process of extracting emotions from user's posts by processing unstructured texts and preparing models that extract knowledge from it. In this study, we consider Twitter; one of the prominent social network sites, to analyze the upcoming 2023 Nigeria election. Given the statistics, Twitter has an active monthly user of 316 million and, on the average, about 500 million tweets are posted daily. A review of related works in subsequent section shows that Twitter is one of the most powerful tools in political analysis. In the current fast-paced global network system, information spreads digitally between users and shapes the way these users feel about an event, thereby making it crucial to understand the thought polarity, emotions and sentiment of the masses.

BERT (Bidirectional Encoder Representations from Transformers) is a powerful natural language processing (NLP) model that has been widely used for sentiment analysis, which is the task of determining the sentiment or emotional tone of a piece of text, such as a review or a tweet [11,12]. Some advantages of using BERT for sentiment analysis include contextualized representations, robust pre-training capability, bidirectional encoding, fine-tuning capability, ability to handle long-range dependencies as well as state-of-the-art performance [13,14]. BERT has been documented to outperform several classical machine and deep learning models [15,16]. This study has been conducted to understand opinions on Nigeria 2023 presidential election using Twitter dataset. It aims to capture, process and evaluate the public opinion from three main perspectives: sentiment and timeline analysis of the personal accounts of contesting candidates; sentiment and general tweet analysis of the public on the three candidates and sentiment and general tweet analysis of the public on the Nigeria 2023 elections. The study would therefore concentrate on the following methodology:

i. Identifying keywords, hashtags and accounts which wholistically explain the subject matter as well as capture the top three contestants for Nigeria 2023 presidential elections.
ii. Scraping the tweets through Twitter API using Python programming.
iii. Data cleaning (removing white spaces, links, punctuations, stop words, tokenization, retweet).
iv. Developing three machine learning models (LSTM, BERT and LSVC) and training with existing annotated IMDB dataset.
v. Using Natural Language Understanding techniques such as sentence polarity, topic modeling, entity extraction, word frequency, word cloud etc. to understand the personal profiles of the three candidates.
vi. Analyzing the result to predict the direction of the election to be conducted in 2023.

The study is further structured into sections: the first section discusses existing works related to our study; the next section which covers methodology explains in detail the technique, models construction and evaluation as well as other analyses done in this to achieve our main aim and objectives, the next section discusses the results obtained in the various experimental setups while, finally we discuss the results and concludes with our findings and direction for future work.

## 2 Related works

Sentiment analysis has been used to predict the opinions of the citizens on US election using Twitter data [17]. The authors used 17,000 tweets to train their model (Naïve Bayes) and the model achieved a less than 60% prediction accuracy by classifying the tweets into positive, negative, neutral and not-sure and this assisted in analyzing real time tweets from the people which gave great insights about public opinions on each candidate. Another study [18] used Twitter dataset to analyze tweets to get international opinions concerning a protest that happened in India conducted by the farmers and about 20,000 tweets was scraped to analyze and categorize tweets into positive, negative and neutral. Bag of words and TF-IDF were used to conduct the analysis and Bag of words outperformed TF-IDF. Other authors [19,20] also established that Twitter can be used as an election indicator and has the ability to predict the favorite candidate of the people to emerge as the winner before the election is conducted. The people gave positive opinions about Donald Trump in almost all states in the United States prior to election. 1,000,000 tweets were collected from various users from different states and sentiment analysis was conducted. A study [21] used Twitter data to check and conduct how different countries affected by the Corona virus coped with the situations. Tweets posted in English were analyzed to give the opinion and emotion of the people concerning the pandemic in their respective countries and 50,000 tweets were used in the study.

Studies combined different features and used ensemble models to increase the detection of polarity of tweets for sentiment analysis and established that unsupervised and ensemble machine learning models outperformed other classical machine learning models in detecting opinions from text [22,23]. Authors have used Twitter data to examine political homophily in American Presidential Elections in 2016 where 4.6 million tweets were collected for analysis [24].

In some studies, authors used the ratio of positive message rate and negative message rate to predict the likely winner of a forthcoming election using twitter data and it showed that these opinions could be used to predict candidate that will emerge as the winner [25]. Twitter data has been used to establish that social media is not only used to express opinions, but it is also used to share ideas and opinions among other users. Authors used 100,000 tweets to predict German federal election in 2009 which could serve as a political indicator for the election [26] and another study [27] also predicted the outcome of German presidential election of 2021 using 58,000 tweets which they established that traditional machine learning methods like Naive Bayes performed less than transformer-based models like the bidirectional encoder from transformers (BERT).

Authors [28] performed social media sentiments about political parties to study and forecast Pakistan's general election. They used supervised machine learning algorithms to classify tweets into positive, negative, and neutral. The findings of their experiment show that social media content can be a useful indication for identifying political behavior of various parties. In another study [29], 90154 tweets were analyzed and the results were compared with the actual election results, their model predicted the winning party accurately.

Our overall goal in this study is to determine the sentiments in tweets with mentions of election-related words for the upcoming Nigeria 2023 elections and find if these tweets can provide meaningful insights regarding the election outcome. Some relative strengths have been identified from this study:

i. Size of dataset: It is noteworthy that bigger datasets enhance NLP models and improve their performance [30]. Having as large as two million tweets will enhance the statistical and predictive credibility of this study and also gives a more comprehensive view of the discourse.
ii. Further NLU tasks such as topic modeling, tf-idf, context-based word-cloud, etc. help to provide a better applicability of the study vis-à-vis the candidates and their impressions.
iii. Social network analysis (SNA) [31] is another strength of this study. This sees impression beyond the ones created by the candidates. It further analyses the network of verified friends around the candidates and their related activities towards their favorite candidates. Conducting SNA in this study for each respective candidate helps in determining homophily, assortativity, associativity, multiplexity and mutuality in the network of prominent friends of each candidate.
iv. Further insights from the personal activities of the candidates were also used to measure their respective winning tendencies vis-à-vis tweet pattern analysis, impression analysis, sentiment analysis of personal tweets etc. This is not prominently considered in the previous works as evident in the reviewed literature.
v. Timeliness is another strength of this study as this study pre-dates the actual election.

## 3 Methodology

This study seeks to analyze tweets of the political discourse around the upcoming 2023 Nigeria presidential election and its prominent contesting candidates and this section describes in detail the approach used in discovering the sentiments of people around this area of public interest. Fig. 1 depicts the framework used in the tweet analyses done in this study. Every tweet with a political content either contains a neutral, positive or negative sentiment for or against a party or candidate. The sentiments contained in tweets especially when it is specific to a candidate is not easy to compute with algorithms since emotion expression varies with the personality, region and cultural background of each person. Since this is an unstructured (unlabelled) dataset, sentiment analysis is often challenging because of the features, context and semantics peculiarity of each tweet.

**Fig. 1:** Framework for twitter-based NLP analysis for Nigeria 2023 elections.

This process started with identification of tweets, trends, keywords and hashtags which wholistically represents the discourse around Nigeria 2023 elections. This is used in a logical structure to scrape tweets from Twitter. The tweets are grouped into the personal tweets of each candidate and the general tweets of the public about the election. The preprocessed dataset was passed into our NLP pipeline to detect sentiments in the posts which is in turn used to perform analyses and provide insights concerning the election.

### 3.1 Dataset

A total of 2,059,113 raw tweets was extracted [32] over a period of four months (June to September 2022). This was collected using tweepy [33], an open-source python library to access the Twitter API using the provided authorization and access tokens. The chosen start date is justified by the fact that the declaration of intent to contest for Presidency began fully in June 2022. The exact search terms used for scraping was carefully constructed to capture tweets about each of the three candidates as well as the general view on the upcoming elections. The dataset contained 360387 unique users from 27 uniquely identifiable countries and the attributes are described in Table 1. Only tweets in English were considered for this study.

**Table 1:** Feature description of dataset.

Feature	Description
TweetId	Unique identifier for each tweet
TweetDate	Date tweet was posted
Username	Twitter handle of the poster
Tweet	The twitter post
UserLocation	Coordinates (if available) of user
UserVerifiedStatus	True if the post is from a Twitter-verified account and False otherwise
UserFollowerCount	Number of followers the user has
FollowingCount	Number of accounts the user follows
AccountCreationTime	The date the user joined Twitter
TweetLocation	Location name of where the tweet was posted
ReplyCount	Number of replies of the tweet
FavoriteCount	Number of likes of tweet
Retweet	Number of retweets

### 3.2 Data preprocessing

To fully prepare the scraped dataset for computation and to reduce bias in the sentiment models, the dataset was preprocessed to remove noisy, inconsistent and irregular patterns [34]. The tweets were originally unstructured and unlabelled, full of noise, unwanted texts and emojis. In this study, the preprocessing was done in a precise and systematic manner as given in Algorithm 1. Our data cleaning approach also included duplicates removal, @-mentions removal, RT which implies retweet and hashtag removal, since all these essentially do not affect the sentiment of the actual tweet.

Algorithm 1 Algorithm for Preprocessing our Twitter Dataset

**Table:** 

Input: Twitter comments or text data Output: Pre-processed text data
For each comment in the Twitter data file Initialize temporary empty string processedTweet to store result of output. 1. Replace all URLs or https://links with the word ‘URL’ using regular expression methods and store the result in processedTweet. 2. Replace all ‘@username’ with the word ‘AT_USER’ and store the result in processedTweet. 3. Filter All #Hashtags and RT from the comment and store the result in processedTweet. 4. Look for repetitions of two or more characters and replace with the character itself. Store result in processedTweet. 5. Filter all additional special characters (: n | [ ] ; : {} – +(.)< > ? ! @ # % *) from the comment. Store result in processedTweet. 6. Remove the word ‘URL’ which was replaced in step 1 and store the result in processedTweet. 7. Remove the word ‘AT_USER’ which was replaced in step 1 and store the result in processedTweet. Return processedTweet.

To fully achieve this algorithm, we leveraged on Python's string manipulation, pattern and regular expressions capabilities such that, as a result, the filtered data can achieve high performance in analyzing data when the machine learning algorithm is applied. With the knowledge that there are unrelated tweets with just anchor tags of the election trend, the data was further checked for the initial keywords of interest and unmatched tweets were eliminated. The final dataset is then separated into personal tweets of the candidates and public tweets. The processedTweet was then tokenized. Tokenization is a term which describes separating a corpus into smallest, syntactically meaningful, units. It is a fundamental step in modeling text data which aids in understanding the meaning behind the text by analyzing the sequence of the words. Porter stemmer was used to reduce the inflection towards their root forms. This was done by stripping the suffix to produce stems [35]. This is then passed into the NLP pipeline for processing.

### 3.3 Natural language processing (NLP) and Natural Language Understanding (NLU) tasks

Natural Language Processing (NLP) and Natural Language Understanding (NLU) describe a comprehensive set of standard tasks and techniques for automatic generation, manipulation and analysis of natural human languages [36]. These enable us to process a huge amount of unstructured corpus through sentence- and token-based analysis as well sentence- and document-level polarity via state-of-art linguistic and lexical processing tools such as WordNet, SentiWordNet and Treebanks [[37], [38], [39]]. The NLP techniques involved in this study include word tokenization, word stemming and lemmatization, topical modeling, named-entity recognition, summarization, word cloud, sentiment analysis and keyword extraction.

a. *Word Tokenization:* The raw tweets after preprocessing and cleaning is broken down into smallest recognizable words and punctuations known tokens [40], the goal of which is generate the list of words which eventually is used for word cloud, summarization and sentiment analysis. The accuracy of this task is often influenced by the training vocabulary, unknown words and out-of-vocabulary (OOV) words.
b. *Stemming and Lemmatization:* This transforms our tokens to its base – dictionary – form by filtering the affixations or by changing a vowel from the word [41]. Stemming and lemmatization aim to reduce the inflectional forms of a word and occasionally related derivational forms to a root form.
c. *Topic Modeling:* Topic modeling is a technique for unsupervised categorization of the twitter documents which helps to identify natural groups of words even when we are not certain what the outcome will be. This gives us a general understanding of the discourse around our corpus. In this study, we used the Latent Dirichlet Allocation (LDA), a particularly popular algorithm for achieving this task [42,43]. A n− dimensional Dirichlet random variable θ takes values in the (k−1)-simplex, that is, a k-vector θ lies in the k−1 simplex iff $\theta_{i}\geq 0,\Sigma_{\left\{i=1\right\}}^{k}\theta_{i}=1$ and has the probability density function on this simplex as given in Equation (1)

(1) $$p\left(\theta |\alpha \right)=\frac{\Gamma \left(\Sigma_{\left\{i=1\right\}}^{k}\alpha_{i}\right)}{\Pi_{i=1}^{k}\Gamma \left(\alpha_{i}\right)}\theta_{1}^{\left\{\alpha_{1}-1\right\}}\ldots \theta_{k}^{\left\{\alpha_{k}-1\right\}}$$

where α is a k− vector with component $\alpha_{i}>0$ and Γ(x) is the Gamma function.

*d. Word Cloud:* We used WordCloud, also called TagCloud to visually represent our Twitter corpus. Tags are tokens, the importance of which is represented with font size or color as a depiction of word significance and word co-occurences. The size of each word in our WordCloud is given in Equation (2).

(2) $$s_{i}=\left\lceil \frac{f_{\max}\cdot \left(t_{i}-t_{\min}\right)}{t_{\max}-t_{\min}}\right\rceil \forall t_{i}>t_{\min}\;else\;s_{i}=1$$

where $s_{i}$ is display font size

$f_{\max}$ is the maximum font size

$t_{i}$ is the count

$t_{\min}$ is the minimum count

$t_{\max}$ is the maximum count

Words in our WordCloud appear bigger the more often they are mentioned and are great for visualizing unstructured text and getting insights on trends and patterns [44,45].

e. *Sentiment Analysis:* We used sentiment analysis as a core component of this study. Sentiment analysis, often regarded as opinion mining, is a natural language processing (NLP) method for identifying the positivity, negativity, or neutrality of data. We used sentiment analysis on our processed textual data to track the perception and reviews of twitter users as regards each of the three prominent contestants of the Presidential election and to summarize the view of the masses in general. A tokenized tweet is sent to our prediction models for processing and its performance was measured. LSTM, a complex area of deep learning, belongs to a class of Recurrent Neural Network (RNN) which can learn order dependence in sequence prediction class of problems [[46], [47], [48]]. This behavior is essential for solving complicated problems in areas like speech recognition and machine translation, among others.

. The proposed LSTM model used in this study is divided into three layers: the tokenize layer, the sigmoid layer and the output layer. The *tokenize* layer has been achieved outside the LSTM model. The LSTM layer is defined by the hidden state dimensions and number of layers. The full connected layer maps the output of the LSTM layer to a desired output size. The sigmoid layer is the activation layer which turns all output values into the map from a closed and bounded interval [−1,1] while the output, the final layer, gives the probability score.

The Bidirectional Encoder Representations from Transformers (BERT) model is a Google AI Language masterpiece which has been widely applied in a wide range of NLP tasks [49,50]. The main strength of the BERT model is its application of bidirectional training of Transformer which is a popular attention model to language modeling. Earlier similar models looked at text sequences from either a left-to-right or a combined left-to-right and right-to-left training perspective. BERT models have demonstrated that bidirectionally trained language models can comprehend context and flow of language more deeply than single-direction language models [51]. Classification tasks such as sentiment analysis are done similarly to Next Sentence classification, by adding a classification layer on top of the Transformer output for each token. The Linear Support Vector Classifier was used to test the accuracy of our deep models. SVM has been one of the most robust prediction techniques which is based on a statistical learning framework [52]. Its workings and model development strategies have been broadly explained in some existing works [[53], [54], [55]].

Table 2 shows the configuration of our models where applicable. For BERT model, we started with a pretrained model where English language was used as for masked language modeling (MLM). This helped to remove noise, unify case sensitivity and correct spelling errors. During modeling, the dataset was chunked into a single train-test sample with Adam Gradient Optimizer with a learning rate of 5e-07 and numerical stability constant of 1e-08. We avoided overfitting and bias by using a dropout layer with dropout probability of 0.4. Being a pretrained model, we used a training time of 10 epochs. For LSTM and LSVC, we set the parameters for each layer as shown in Table 2.

**Table 2:** Configurations of the sentiment models.

Model	Layer	Output Shape	Parameters
LSTM	Input (Word Embedding) Layer	32	2643772
	Hidden Layer 1	64	23844
	Hidden Layer 2	64	3892
	Output Layer	1	65
BERT	–	–	109482240
LSVC	–	–	–

The sentiment models were assessed using accuracy, area under curve (AUC), recall, false positive rate (FPR), precision and F-measure as seen in Equations (3)–(7). The area under the ROC curve (AUC) is a plot of true positive rate (TPR, or specificity) against false positive rate (FPR, or sensitivity). The true positive rate (TPR), sensitivity, or recall is the number of sentiment labels predicted positive that are actually positive. Recall is defined by Equation (4). The false positive rate (FPR) is the number of sentiment labels predicted positive that are actually negative and is defined in Equation (5). Precision is the proportion of the predicted positive cases that were correct. The precision can be calculated using Equation (6). The F-Measure score is the harmonic mean of the precision and recall. This evaluates the equivalency between the sensitivity (recall) and the precision (correctness) of the data. This gives us the interpretation of how the measure recall and precision values behave for the dataset. The F-measure can be calculated using Equation (7).

Let $TP_{+}$ = true positive for all positive tweets, $TP_{-}$ = true positive for all negative tweets, $TP_{\varphi }$ = true positive for all neutral tweets. Then:

(3) $$Accuracy=\frac{TP_{+}+TP_{-}+TP_{\varphi }}{\Sigma all\;instances}$$

(4) $$TPR,Sensitivity,Recall=\frac{\Sigma TP_{+}}{\Sigma All\;Actual\;Positives}$$

(5) $$FPR=\frac{\Sigma TP_{-}}{\Sigma All\;Actual\;Negatives}$$

(6) $$Precision=\frac{TP}{TP+FP}$$

(7) $$F-Measure=\frac{2*Precision*Recall}{Precision+Recall}$$

## 4 Experimental setup

In this study, we were interested in what goes on in the Twitter space as regards the upcoming Nigeria's 2023 elections. We sought to achieve this via scraping of tweets concerning the prominent aspirants, the election in general as well as through the analysis of the personal tweets of the aspirants. For these individual datasets, we analyzed their tweet sentiments, tweet frequency, tweet popularity, hashtag and wovrd tag outputs as well as their opinion polarity. This helped to gain understanding of the relative social media power of each candidate, their strategies, strengths, weaknesses, opportunities and threats of each of the three candidates. We also performed social network analysis of the social media circles of friends kept by each of the candidates. Sentiment analysis gave the perspective of each tweet, WordCloud gave a summarization of entities concerning them while social network analysis showed the connections maintained by each of the candidates. Personal and public tweet analyses give understanding of trends, patterns, keywords and sentiments of each candidate as well as the masses respectively. In building and validating our sentiment model, we used the IMDB dataset which contained 50000 movie reviews and has widely been used for sentiment analysis tasks [56]. We passed the preprocessed IMDB dataset into our LSTM, BERT and LSVC models and compared their accuracies. We then passed our preprocessed Twitter dataset into the pre-trained models. The performance of our models on the IMDB dataset is our confidence in the sentiments returned for each tweet in this study.

## 5 Results

### 5.1 Dataset

Our Twitter dataset was extracted from June 1 to September 30, 2022 containing tweets related to the candidacies of Tinubu, Atiku and Obi and generally about the upcoming 2023 Nigeria Presidential elections. There is a global interest in the upcoming Nigeria 2023 elections from many prominent countries of the world including Nigeria, United States of America, United Kingdom, Canada, Germany and Dubai. Table 3 shows the statistics of the countries with the highest tweets. The location of majority of users are marked as Not Available (NA).

**Table 3:** Tweets by countries.

Countries	Number of Tweets
*Nigeria*	873,111
*USA*	45,918
*UK*	30,042
*Canada*	17,898
*Others*	230,229
*NA*	861,915
*Total*	2,059,113

### 5.2 Sentiment analysis model performance

Three models were used in this study and their performance was measured. Table 4 shows the performance for the models which were developed to determine the sentiments in the datasets. The BERT model gave the best prediction with the highest accuracy, AUC, precision, recall and F-Measure. The BERT model, however, spent the most time in its model building and predictions with batch size of 64. This is because it is a deep neural network model with a deeper intermediate layer. The result shows that BERT model outperformed the other two models with a recall of 0.925, precision of 0.827, F-Measure of 0.829, accuracy of 0.880 and AUC of 0.876.

**Table 4:** Performance of the models using the IMDb dataset with batch size of 64.

	Recall	Precision	F-Measure	Accuracy	AUC	Processing Time(s)
LSTM	0.872	0.827	0.829	0.88	0.876	122
SVC	0.764	0.814	0.792	0.73	0.812	95
BERT	0.925	0.885	0.917	0.94	0.947	322

### 5.3 Personal tweet analysis

In this section, we examined the personal Twitter accounts (@atiku, @officialABAT and @PeterObi) of each of the candidates. The first dataset contained the personal tweets of the candidates and Table 5 shows their tweet summarization, tweet frequency and impressions made by their personal tweets. It shows that Atiku joined tweeter the earliest but highest tweets during the time covered by this study was from Peter Obi. Peter Obi came first in total number of retweets, mentions and favorited tweets. Atiku, however, has the highest number of followers.

**Table 5:** Personal tweet summaries of the presidential candidates.

*Handles*	Atiku Abubakar	Peter Obi	Tinubu
	@atiku	@peterobi	@officialABAT
Total Tweets	6,654	1,226	2,156
Tweet since June 1st – September 30th^,^ 2022	490	753	199
Total Retweet	2,233,022	3,096,402	304,607
Tweet Retweet June 1st – September 30th^,^ 2022	189,493	2,444,221	117,452
Total Favorited	7,557,994	11,685,304	1,036,233
Tweet Favorited June 1st – September 30th^,^ 2022	904,423	9,396,626	546,369
Number of Followers	4,592,032	2,211,370	1,458,411

The sentiment analysis of tweets posted by the three candidates is summarized in Table 6. Fig. 2 shows the sentiment analysis of the favorite words of the candidates. It shows that Peter Obi has more favorite words as well as more positive favorite words than either of his peers.

**Table 6:** Personal tweet sentiments.

	Atiku Abubakar			Peter Obi			Tinubu		
	Negative	Neutral	Positive	Negative	Neutral	Positive	Negative	Neutral	Positive
All Tweets	696	3,920	2,035	109	803	312	309	1368	477
Tweets Since June 1 – September 31	34	346	110	59	537	156	6	126	67
Total Favorited Tweets Since June 1 – September 31	33,549	593,389	277,485	653,356	6,385,453	2,353,280	7,262	398,440	140,667
Total Retweeted Tweets Since June 1 – September 31	7,853	137,640	44,000	183,661	1,729,385	529,879	1,429	91,078	24,945

**Fig. 2:** Sentiments of the favorite words of the three candidates.

Fig. 3, Fig. 4 depict the flow of tweets of each candidate on a weekly and yearly basis. The daily tweet pattern shows that Atiku tweets most on Thursdays, while Tinubu and Peter Obi tweets most on Wednesdays. The hourly tweet pattern shows that Atiku and Peter Obi spend the early hours of the day tweeting while Tinubu tweets in the afternoon around 2pm and 7pm. The yearly pattern shows that Peter Obi has not been active on Twitter until the year he started vying for the seat of Presidency. However, a similar pattern is evident with Atiku and Tinubu who tweet most only during election years.

**Fig. 3:** Daily tweet pattern of the Presidential candidates.

**Fig. 4:** Yearly tweet pattern of the Presidential Candidates.

Fig. 5, Fig. 6, Fig. 7 show the word clouds of the favorite words, mentioned users and popular hashtags of the three vying candidates. These figures reveal that Atiku was big on words such as Nigeria, government, family, health and democracy; Peter Obi is frequent with words such as Nigeria, government, economy, leadership, diaspora, education, security, etc. while Tinubu's tweets are centered around Nigeria, people, government, party and Buhari. Fig. 7 shows that Atiku and Peter Obi used hashtags of their tours to various locations particularly local and international places respectively while Tinubu prefers to use Colloquium, ReadytoLead and ReadytoServe.

**Fig. 5:** WordCloud of the favorite words of the Presidential Candidates.

**Fig. 6:** WordCloud of the mentioned users in tweets of the Presidential Candidates.

**Fig. 7:** WordCloud of the mentioned hashtags in tweets of the Presidential Candidates.

The mentioned hashtags show that Atiku showcases his travels to some non-Northern states such as Bauchi, Enugu, Oyo, Osun etc. and is an advocate of *#oneNigeria* as part of his campaign strategies. Peter Obi seems to be an international traveler with visits to Texas, Michigan, Washington DC, Havard, Atlanta etc. He also traveled to Jos as part of his campaign to voters outside his territory. Tinubu, although may have strategies outside the Twitter space, is not clear in his tour and campaign zone strategies.

Our social network analysis on each of the three candidates for the period covered in this study produced Fig. 8. This was used understand the Twitter activities of the verified friends of the Presidential candidates in terms of retweets and mentions. It shows that Tinubu maintained the strongest and most active verified network of Twitter friends, followed by Peter Obi. Atiku, on the other hand, has many friends who are dormant and inactive to his posts. Tinubu has prominently active verified friends including the incumbent President Muhammadu Buhari, Babatunde Raji Fashola (minister for Works and Housing of Nigeria), Babajide Sanwoolu (current Governor of one of the most populous states in Nigeria) etc. Atiku has @RenoOmokri as a very strong and active member. Peter Obi has more networks than Atiku but less than Tinubu.

**Fig. 8:** Social network of the presidential candidates.

### 5.4 Public tweet analysis

The public tweets concerning Atiku, Peter Obi and Tinubu were analyzed to obtain their respective public opinions. Table 7 shows the tweet summaries of the public tweets as obtained in this study while Table 8 shows the result of sentiment analysis of the public tweets categorized into each of the three candidates and Fig. 9 shows the overall sentiments of the masses concerning these candidates.

**Table 7:** Public tweet summaries of the presidential candidates.

	Atiku Abubakar	Peter Obi	Tinubu
Search Term	ATIKU OR ATIKULATED	PETER OBI OR OBIDIENT	TINUBU OR JAGABAN OR BATIFIED
Tweet since June 1st – September 30th^,^ 2022	50,688	980,336	1,028,058
Tweet Retweet June 1st – September 30th^,^ 2022	444,903	5,122,375	5,265,670
Total Favorited June 1st – September 30th^,^ 2022	1,366,512	17,784,008	16,430,587

**Table 8:** Summarization of public tweet sentiments.

	Atiku Abubakar			Peter Obi			Tinubu		
	Negative	Neutral	Positive	Negative	Neutral	Positive	Negative	Neutral	Positive
Tweets Since June 1 – September 31	6,599	33,960	10,105	35898	457,019	504,665	894,766	409,643	587,993
Total Favorited Tweets Since June 1 – September 31	162,497	1,026,372	177,438	1,150,954	6,976,112	8,008,726	1,765,443	4,004,534	9,309,876
Total Retweeted Tweets Since June 1 – September 31	53,120	348,001	43,729	534,775	1,856,223	2,998,766	859,882	2,034,598	2,650,986

**Fig. 9:** Overall opinions based on public tweets.

## 6 Discussion

This work is primarily focused on the analysis of the Twitter space as regards the discourse around Nigeria 2023 presidential elections. We took it further by, first, analysis the individual tweets of the three candidates as well as the public opinion about them. The aim is to generate insights on each candidate and discover their strengths and weaknesses as well as suggest areas of improvements regarding their road to Aso-Rock. Our major analysis was centered on tweets on the election vis-à-vis sentiments expressed, frequently mentioned terms and impressions via mentions, favoriting and retweets. We observed that three candidates have their specific strategies and positives:

i. Atiku concentrates more on local networks and conferences.
ii. Peter Obi recently recognized the Twitter space as a viable medium of manifesto in recent times and keyed into it. He also has the most international outfits of the three candidates.
iii. Tinubu is a network strategist who maintained an active Twitter network. This will help in creating a ripple effect of his campaign strategies.
iv. Peter Obi leads in the overall impressions and engagements since the three candidates declared their intents to run. He owns the highest tweets, retweets, mentions and favorited count among the three electorates.

It is interesting, but somewhat disappointing, to note that the three candidates did not pay enough attention to discussing the power, unemployment, education and security of the nation. As at the time of this writing, there is a chaotic dwindling of the nation's economy, University education has been shut down for nine months, there has been an epileptic power supply due to incessant collapse of the national grid and the security system has not found solution to bombings, killings and kidnappings across the Federation. This, indeed, should be the major campaign points of each of these candidates; but unfortunately, not. The tweet frequency and total impressions of the public tweets concerning the three candidates say a lot.

Our exploratory data analysis reveals that while Twitter is a good platform for political discussion and debate, a very small percentage of people control it. Also, majority of Twitter users (who disclosed their geo-location) only use Twitter to follow trends and conversations. During the height of the declaration of intent to run for presidency, it appears that most users who published their geolocation are passive and do not actively participate in dialogues nor express their opinions.

One strength of this work is that sentiment analysis and NLP, to the best of our knowledge, has not been applied to understand elections in Nigeria. This shows that this work is novel in the Nigerian context. Another strength is the fact that most works do not consider the personal profiles of the candidates they examine. In this work, we provide an omnibus study which wholistically examines the internal and external profiles of the candidates to project a clearer and more reliable picture of the forthcoming Presidency election. Also, most studies in the past were conducted retrospectively. We, in this work, conducted a scientific study prior to the election and present the result as is. This means that this study is independent and bias-free. Social network analysis on Twitter profiles were uncommon in reviewed works. In this study, we understood each candidate in the light of the friends they keep on the social media space. Finally, the size of our dataset is a major relative advantage to existing works. Authors took time to scrape the data comprehensively which necessarily and sufficiently covers Twitter discourse on the subject matter from the declaration of intent to run to the date this study was closed.

One limitation of this study is the time covered in the study. Although three months gave a very huge number of tweets, we know that strategies of campaign and manifestoes may change as events unfold. Since the result of the actual election outlive this study, we may not have a sufficient ground truth to validate the results of our experiments. Another limitation is that majority of eligible voters may not have Twitter accounts or contribute to the online election discourse. This may have a lot to say about comparing the outcome of the results in this study with the actual results of the actual election, come 2023. Although the authors attempted to further classify the sentiments by states using geocordinates, we were limited by the fact that most users prefer not to share their locations for obvious reasons.

## 7 Conclusion and future work

Social media platforms have proven to be an excellent tool which gives us opportunities to share thoughts, idea and opinions. Due to the upsurge in the number of internet users, social media networks have grown in popularity. As a result, there has been a tremendous increase in the quantity of tweets from individuals who expressed their opinions about the Nigeria 2023 elections all over the world. Users have shown their personal agitation on this discourse.

Finally, it is noteworthy in our candidate analyses that:

i. Peter Obi leads the chart in terms of Twitter impressions and engagements.
ii. Tinubu shows the strongest connection of active friends. This is a hidden winning strategy towards the presidential election.
iii. Atiku, although with the most followers, made the least impression on Twitter.
iv. If Nigeria 2023 presidential election is a two-horse race (as in Table 2), then Tinubu and Peter Obi are the real candidates to beat in the forthcoming presidential race.

In this work, we have investigated scientific and analytical methods for understanding the opinion polarity of people by developing a sentiment analysis model and determining the course that the Nigeria 2023 election campaign is taking. We found the relative strengths and weaknesses of each candidate and presented them as is. This study will be helpful for each candidate in consolidating their strengths and intensifying efforts where they lag. Although LSTM, a class of deep neural network, is a powerful tool in NLP [57,58], future work may look at applying other sentiment classification models for polarizing the public opinions.

We conclude that opinion mining from Twitter can form a general basis for generating insights for election as well as modeling election outcomes. Overall, sentiment analysis can offer several advantages for election prediction, including real-time data, large-scale data analysis, unbiased insights, early warning signals, cost-effectiveness, and complementarity with other methods. By leveraging the power of state-of-the-art natural language processing and text analysis, sentiment analysis can provide valuable insights into public sentiment, helping predict election outcomes more accurately.

## Author contribution statement

All authors listed have significantly contributed to the reported implementation, development and writing of this article.

## Data availability statement

Data will be made available on request.

## Declaration of competing interest

The authors declare that they have no known competing financial interests or personal relationships that could have appeared to influence the work reported in this paper.

## References

[1] Roberts M.E. (2018). What is political methodology?. PS Political Sci. Polit..

[2] Achen C.H. (2002). Toward a new political methodology: microfoundations and ART. Annu. Rev. Polit. Sci..

[3] Ascher W. (1982). Political forecasting: the missing link. J. Forecast..

[4] Remmer K.L. (1993). The political economy of elections in Latin America, 1980–1991. Am. Polit. Sci. Rev..

[5] Oluro M.J., Bamigbose J.O. (2021). Legislative cross-carpeting, multiparty system and the challenges of democratic good governance in Nigeria. J. Publ. Adm. Govern..

[6] Cameron M.P., Barrett P., Stewardson B. (2016). Can social media predict election results? Evidence from New Zealand. J. Polit. Market..

[7] Seurin P. (2022). H2-golden-retriever: Methodology and tool for an evidence-based hydrogen research grantsmanship. arXiv preprint arXiv:2211.08614.

[8] Allcott H., Gentzkow M. (2017). Social media and fake news in the 2016 election. J. Econ. Perspect..

[9] Hendricks J.A., Schill D. (2017).

[10] Wani G., Alone N. (2014). A survey on impact of social media on election system. Int. J. Comput. Sci. Inf. Technol..

[11] Gao Z. (2019). Target-dependent sentiment classification with BERT. IEEE Access.

[12] Munikar M., Shakya S., Shrestha A. (2019). 2019 Artificial Intelligence for Transforming Business and Society (AITB).

[13] Malte A., Ratadiya P. (2019). Evolution of transfer learning in natural language processing. arXiv preprint arXiv:1910.07370.

[14] Zaheer M. (2020). Big bird: transformers for longer sequences. Adv. Neural Inf. Process. Syst..

[15] Sun C., Huang L., Qiu X. (2019). Utilizing BERT for aspect-based sentiment analysis via constructing auxiliary sentence. arXiv preprint arXiv:1903.09588.

[16] Li X. (2019). Exploiting BERT for end-to-end aspect-based sentiment analysis. arXiv preprint arXiv:1910.00883.

[17] Wang H. (2012). Proceedings of the ACL 2012 System Demonstrations.

[18] Neogi A.S. (2021).

[19] Somula R. (2016). Smart Intelligent Computing and Applications. 2020.

[20] Chandra R., Saini R.J.I.A. (2021).

[21] Kausar M.A. (2021).

[22] Carvalho J., Plastino A.J.A.I.R. (2021).

[23] Bibi M. (2022).

[24] Caetano J.A. (2018).

[25] Yavari A. (2022).

[26] Tumasjan A. (2010). Proceedings of the International AAAI Conference on Web and Social Media.

[27] Schmidt T. (2022). Proceedings of the 18th Conference on Natural Language Processing.

[28] Razzaq M.A., Qamar A.M., Bilal H.S.M. (2014). 2014 IEEE/ACM International Conference on Advances in Social Networks Analysis and Mining (ASONAM 2014).

[29] Singh P., Sawhney R.S., Kahlon K.S. (2017). International Conference on Advanced Informatics for Computing Research.

[30] Roberts K. (2016). Proceedings of the Clinical Natural Language Processing Workshop.

[31] Freeman L. (2004). The development of social network analysis. Study Sociol. Sci..

[32] Al Walid M.H., Anisuzzaman D., Saif A.S. (2019). Data analysis and visualization of continental cancer situation by Twitter scraping. Int. J. Mod. Educ. Comput. Sci..

[33] Kusumasari B., Prabowo N.P.A. (2020). Scraping social media data for disaster communication: how the pattern of Twitter users affects disasters in Asia and the Pacific. Nat. Hazards.

[34] Hemalatha I., Varma G.S., Govardhan A. (2012). Preprocessing the informal text for efficient sentiment analysis. Int. J. Emerg. Trends Techn. Comp. Sci.(IJETTCS).

[35] Jivani A.G. (2011). A comparative study of stemming algorithms. Int. J. Comp. Tech. Appl.

[36] Cambria E., White B. (2014). Jumping NLP curves: a review of natural language processing research. IEEE Comput. Intell. Mag..

[37] Fellbaum C. (2010). Theory and Applications of Ontology: Computer Applications.

[38] Baccianella S., Esuli A., Sebastiani F. (2010). Proceedings of the Seventh International Conference on Language Resources and Evaluation.

[39] Taylor A., Marcus M., Santorini B. (2003).

[40] Mielke S.J. (2021). Between words and characters: a brief history of open-vocabulary modeling and tokenization in nlp. arXiv preprint arXiv:2112.10508.

[41] Lovins J.B. (1968). Development of a stemming algorithm. Mech. Transl. Comput. Ling..

[42] Yu H., Yang J. (2001). A direct LDA algorithm for high-dimensional data—with application to face recognition. Pattern Recogn..

[43] Wei X., Croft W.B. (2006). Proceedings of the 29th Annual International ACM SIGIR Conference on Research and Development in Information Retrieval.

[44] Heimerl F. (2014). 2014 47th Hawaii International Conference on System Sciences.

[45] Jin Y. (2017). Development of word cloud generator software based on python. Procedia Eng..

[46] Yu Y. (2019). A review of recurrent neural networks: LSTM cells and network architectures. Neural Comput..

[47] Huang Z., Xu W., Yu K. (2015). Bidirectional LSTM-CRF models for sequence tagging. arXiv preprint arXiv:1508.01991.

[48] Staudemeyer R.C., Morris E.R. (2019). Understanding LSTM--a tutorial into long short-term memory recurrent neural networks. arXiv preprint arXiv:1909.09586.

[49] Devlin J. (2018). Bert: Pre-training of deep bidirectional transformers for language understanding. arXiv preprint arXiv:1810.04805.

[50] Ravichandiran S. (2021).

[51] Lee J.-S., Hsiang J. (2020). Patent classification by fine-tuning BERT language model. World Patent Inf..

[52] Noble W.S. (2006). What is a support vector machine?. Nat. Biotechnol..

[53] Suthaharan S. (2016). Machine Learning Models and Algorithms for Big Data Classification.

[54] Pisner D.A., Schnyer D.M. (2020). Machine Learning.

[55] Widodo A., Yang B.-S. (2007). Support vector machine in machine condition monitoring and fault diagnosis. Mech. Syst. Signal Process..

[56] Tripathi S. (2020). 2020 12th International Conference on Computational Intelligence and Communication Networks (CICN).

[57] Yao L., Guan Y. (2018). 2018 IEEE International Conference of Safety Produce Informatization (IICSPI).

[58] Zhang X., Chen M.H., Qin Y. (2018). 2018 2nd International Conference on Data Science and Business Analytics (ICDSBA).

